# Treadmill Training Increases SIRT-1 and PGC-1**α** Protein Levels and AMPK Phosphorylation in Quadriceps of Middle-Aged Rats in an Intensity-Dependent Manner

**DOI:** 10.1155/2014/987017

**Published:** 2014-06-09

**Authors:** Nara R. C. Oliveira, Scherolin O. Marques, Thais F. Luciano, José R. Pauli, Leandro P. Moura, Erico Caperuto, Bruno L. S. Pieri, Julia Engelmann, Gisele Scaini, Emilio L. Streck, Fabio S. Lira, Ricardo A. Pinho, Eduardo R. Ropelle, Adelino S. R. Silva, Cláudio T. De Souza

**Affiliations:** ^1^Laboratory of Exercise Biochemistry and Physiology, Health Sciences Unit, Extremo Sul Catarinense University (UNESC), 88806-000 Criciuma, SC, Brazil; ^2^Faculty of Applied Sciences, University of Campinas (UNICAMP), 13083-872 Limeira, SP, Brazil; ^3^Post Graduation Program in Motricity Science, Instituto de Biociências, São Paulo State University (UNESP), 13506-900 Rio Claro, SP, Brazil; ^4^Human Movement Laboratory, São Judas Tadeu University, 03166-000 São Paulo, SP, Brazil; ^5^Immunometabolism Research Group, Department of Physical Education, São Paulo State University (UNESP), 19060-900 Presidente Prudente, SP, Brazil; ^6^School of Physical Education and Sport of Ribeirão Preto, São Paulo University (USP), 14040-907 Ribeirão Preto, SP, Brazil

## Abstract

The present study investigated the effects of running at 0.8 or 1.2 km/h on inflammatory proteins (i.e., protein levels of TNF-**α**, IL-1**β**, and NF-**κ**B) and metabolic proteins (i.e., protein levels of SIRT-1 and PGC-1**α**, and AMPK phosphorylation) in quadriceps of rats. Male Wistar rats at 3 (young) and 18 months (middle-aged rats) of age were divided into nonexercised (NE) and exercised at 0.8 or 1.2 km/h. The rats were trained on treadmill, 50 min per day, 5 days per week, during 8 weeks. Forty-eight hours after the last training session, muscles were removed, homogenized, and analyzed using biochemical and western blot techniques. Our results showed that: (a) running at 0.8 km/h decreased the inflammatory proteins and increased the metabolic proteins compared with NE rats; (b) these responses were lower for the inflammatory proteins and higher for the metabolic proteins in young rats compared with middle-aged rats; (c) running at 1.2 km/h decreased the inflammatory proteins and increased the metabolic proteins compared with 0.8 km/h; (d) these responses were similar between young and middle-aged rats when trained at 1.2 km. In summary, the age-related increases in inflammatory proteins, and the age-related declines in metabolic proteins can be reversed and largely improved by treadmill training.

## 1. Introduction

The mitochondrial function impairment in skeletal muscle is one of the physiological limitations of aging [1]. However, there is a considerable variability of aging impact on mitochondrial function [2–6]. Sarcopenia and muscle fatigability in response to aging are associated with the increase of both the reactive oxygen species (ROS) production and the mitochondrial apoptotic susceptibility, as well as the decrease of transcriptional drive for mitochondrial biogenesis [3]. However, the precise underlying mechanisms of these processes remain unclear. Some common regulatory mechanisms that include silent information regulators like sirtuins have been studied [7–9]. The silent information regulator 2 homolog 1 (SIRT-1) may influence the aging processes and many age-associated diseases, including metabolic disorders such as diabetes. SIRT-1 is downregulated in human senescent cells, suggesting that SIRT-1 may be required to extend the replicative life span [10].

Aging processes are orchestrated in part by powerful deacetylators Sirts [7]. For example, the deacetylation of lysine residues of the histone tails by Sirt induces closed chromatin configuration and transcriptional silencing [8]. Besides histone deacetylation, SIRT-1 targets a number of transcription factors such as peroxisome proliferator-activated receptor gamma coactivator-1alpha (PGC-1*α*), which is involved in mitochondrial biogenesis and skeletal muscle differentiation [9, 11]. Thus, SIRT-1-mediated PGC-1*α* deacetylation is a key factor of mitochondrial biogenesis activation [9, 11]. The PGC-1*α* family of regulated coactivators plays a central role in a regulatory network governing the transcriptional control of mitochondrial biogenesis and respiratory function. These coactivators target multiple transcription factors, including nuclear respiratory factors (NRF) 1 and 2 and the orphan nuclear hormone receptor (estrogen-related receptor alpha—ERR*α*), among others [12]. In addition, they themselves are the targets of coactivator and corepressor complexes that regulate gene expression through chromatin remodeling.

The proposed role for PGC-1*α* as a regulator of mitochondrial biogenesis is supported by experiments that verified functional improvements in both cultured cells [12] and transgenic mice [13]. The PGC-1*α* expression is modulated by extracellular signals that control metabolism, differentiation, or cell growth. In addition, in some cases, PGC-1*α* activity is regulated by posttranslational modification by the energy sensors, such as SIRT-1 and AMP-activated protein kinase (AMPK).

AMPK is emerging as a crucial regulator of whole-body energy balance [14]. In skeletal muscle, after being activated, AMPK regulates both the fatty-acid oxidation by the phosphorylation of acetyl-CoA carboxylase (ACC) and the mitochondrial biogenesis by the increase of the expression of vital proteins for proper mitochondrial function, such as citrate synthase and succinate dehydrogenase [15, 16]. In addition, AMPK promotes mitochondrial biogenesis by the increase of both PGC-1*α* levels and other associated mitochondrial proteins [17–20].

The activation of AMPK (e.g., by exercise) triggers an increase in the NAD^+^/NADH ratio, which activates SIRT-1. AMPK also induces PGC-1*α* phosphorylation and primes it for subsequent deacetylation by SIRT-1 [21]. The impact of AMPK and SIRT-1 on the PGC-1*α* acetylation status and other transcriptional regulators will modulate mitochondrial function and activity [21]. In fact, multiple endogenous and exogenous factors regulate mitochondrial biogenesis by PGC-1*α*, SIRT-1, and AMPK, including physical exercise. Physical exercise is known to induce metabolic adaptations in skeletal muscle via activation of these molecules [3, 22]. However, in the aging process, the influence of different training intensities on molecular alterations remains unclear. Thus, this study was designed to test the hypothesis that high training intensity is more effective than low training intensity in restoring SIRT-1, AMPK, PGC-1*α*, and related metabolic enzymes that decrease with aging. Based on the fact that aging is related to increased circulating proinflammatory and lower anti-inflammatory cytokines [23] and knowing that besides the role as an activator of mitochondrial biogenesis, PGC-1*α* also acts as a suppressor of inflammatory cytokines [24], we also investigated the responses of the tumor necrosis factor alpha (TNF-*α*), interleukin 1*β* (IL-1*β*), and nuclear factor kappa-B (NF-*κ*B) to different training intensities in young and middle-aged Wistar rats.

## 2. Materials and Methods

### 2.1. Animals Groups

Male Wistar rats at 2 (young) and 18 (middle-aged) months were used during the experiments. The current investigation followed the university guidelines for the use of animals in experimental studies (protocol number 92/2009). The procedures used in this study received approval from the Research Ethics Committee of Universidade do Extremo Sul Catarinense (Criciúma, Brazil). Young and middle-aged animals were divided into the following groups (*n* = 6): nonexercised (NE), exercised at 0.8 km/h (0.8 km/h), and exercised at 1.2 km/h (1.2 km/h). We selected middle-aged rats in order to study molecular and physiological changes related to mitochondrial function during a life period that still allows preventive actions that can lead to healthy aging. All animals were maintained at temperatures ranging from 20 to 25°C, with a 12-hour light/dark cycle and fed on a standard rodent chow* ad libitum*.

### 2.2. Descriptive Characteristics of Young and Middle-Aged Rats before Exercise Protocols

Before the beginning of the exercise protocols, one set of young and middle-aged rats (*n* = 8) was evaluated for the following parameters: body weight (g), blood glucose (mg/dL), epididymal fat (g/100 g), and serum insulin (ng/mL). The rats were anesthetized with an intraperitoneal (i.p) injection of ketamine chlorohydrate (50 mg/kg; Syntec, Cotia, SP, Brazil) and xylazine (20 mg/kg; Syntec, Cotia, SP, Brazil), and the blood was collected from the cava vein. Serum was separated by centrifugation (1,100 ×g) for 15 min at 4°C and stored at −80°C for further analysis. The epididymal fat was surgically removed, weighted, and expressed as g/100 g of rats' body weight. While rest blood glucose (mg/dL) was measured by a glucometer (Advantage, Boehringer Mannheim, Irvine, CA), the rest serum insulin was determined using a commercially available Enzyme Linked Immunosorbent Assay (ELISA) kit (Crystal Chem Inc., Chicago, IL).

### 2.3. Exercise Protocols

All animals were habituated on a nine-channel motor-drive treadmill (Insight EP 131, Ribeirão Preto, Brazil) at a velocity of 0.6 km/h for 10 min/day during 1 week in order to reduce stress during the training period. The rats did not receive any electric stimulus to run, but manual stimulation was applied. The exercise group performed a running program at constant speed of 0.8 km/h or 1.2 km/h without inclination for 50 min, 5 days per week, during 8 weeks. The nontrained rats were placed on the switched-off treadmill for the same 8 weeks. Forty-eight hours after the last training sessions, the rats were anesthetized with an intraperitoneal (i.p) injection of ketamine chlorohydrate (50 mg/kg; Syntec, Cotia, SP, Brazil) and xylazine (20 mg/kg; Syntec, Cotia, SP, Brazil), and quadriceps was removed for biochemical and immunoblotting analyses.

### 2.4. Protein Analysis by Immunoblotting

The superficial (i.e., rectus femoris composed of type I: 1%, type IIa: 25%, and type IIb: 74%) and deep quadriceps (i.e., vastus intermedius composed of type I: 59%, type IIa: 40%, and type IIb: 1%) [25] were homogenized together in extraction buffer (1% Triton-X 100, 100 mMTris, pH 7.4, containing 100 mM sodium pyrophosphate, 100 mM sodium fluoride, 10 mM EDTA, 10 mM sodium vanadate, 2 mM PMSF, and 0.1 mg of aprotinin/mL) at 4°C (Polytron MR 2100, Kinematica, Switzerland). The extracts were centrifuged at 11,000 rpm at 4°C (5804R, Eppendorf AG, Hamburg, Germany) for 40 min to remove insoluble material, and the supernatants of this tissue were used for protein quantification, according to the Bradford method. Proteins were denatured by boiling in Laemmli sample buffer containing 100 mM DTT, run on SDS-PAGE, and transferred to nitrocellulose membranes. Membranes were blocked, probed, and blotted with primary antibodies. Antibodies used for immunoblotting were antiphospho (Thr172) AMPK, antiphospho (Ser79) ACC, anti-AMPK, and anti-ACC antibodies (Cell Signaling Technology, Beverly, MA, USA); anti-SIRT-1, anti-PGC-1*α*, anti-CPT1, anti-SDH, citrate synthase, anti-Cyt-C, and *β*-actin (Santa Cruz Biotechnology, Santa Cruz, CA, USA); and anti-TNF-*α*, anti-IL-1*β*, and anti-NF-*κ*B (Abcam Biotechnology, Eugene, Oregon, USA). The original membrane was stripped and reblotted with *β*-actin as loading protein. Chemiluminescent detection was performed with horseradish peroxidase-conjugate secondary antibodies (Thermo Scientific, Rockford, IL, USA). Autoradiographs of membranes were taken for visualization of protein bands. The results of the blots are presented as direct comparisons of the area of the apparent bands in autoradiographs and quantified by densitometry using the Scion Image software (Scion Image software, ScionCorp, Frederick, MD).

### 2.5. Activity of Krebs Cycle Enzymes

#### 2.5.1. Citrate Synthase Activity

Citrate synthase activity was assayed according to the method described by Shepherd and Garland [26]. The reaction mixture contained 100 mMTris, pH 8.0, 100 mM acetyl CoA, 100 mM 5,5′-di-thiobis-(2-nitrobenzoic acid), 0.1% triton X-100, and 2–4 *μ*g supernatant protein, and it was initiated with 100 *μ*M oxaloacetate and monitored at 412 nm for 3 min at 25°C.

#### 2.5.2. Succinate Dehydrogenase Activity

Succinate dehydrogenase activity was determined according to the method of Fischer et al. [27], measured by the following decrease in absorbance due to the reduction of 2,6-dichloroindophenol (2,6-DCIP) at 600 nm with 700 nm as the reference wave length (*ε* = 19.1 mM^−1 ^cm^−1^) in the presence of phenazine methosulphate (PMS). The reaction mixture consisting of 40 mM potassium phosphate, pH 7.4, 16 mM succinate, and 8 *μ*M 2,6-DCIP was preincubated with 40–80 *μ*g homogenate protein at 30°C for 20 min. Subsequently, 4 mM sodium azide, 7 *μ*M rotenone, and 40 *μ*M 2,6-DCIP were added, and the reaction was initiated by adding 1 mM PMS and was monitored for 5 min.

### 2.6. Activity of Mitochondrial Respiratory Chain Enzymes

#### 2.6.1. Complex I Activity

NADH dehydrogenase (complex I) was evaluated according to Cassina and Radi [28] by determining the rate of NADH-dependent ferricyanide reduction at *λ* = 420 nm.

#### 2.6.2. Complex II Activity

The activity of succinate-2,6-dichloroindophenol- (DCIP-) oxidoreductase (complex II) was determined using the method described by Fischer et al. [27]. Complex II activity was measured by following the decrease in absorbance due to the reduction of 2,6-DCIP at *λ* = 600 nm.

#### 2.6.3. Complex II-III Activity

The activity of succinate: cytochrome *c* oxidoreductase (complex III) was determined using the method described by Fischer et al. [27]. Complex II-III activity was measured by cytochrome *c* reduction using succinate as substrate at *λ* = 550 nm.

#### 2.6.4. Complex IV Activity

The activity of cytochrome *c* oxidase (complex IV) was assayed according to the method described by Rustin et al. [29] and measured by following the decrease in absorbance due to the oxidation of previously reduced cytochrome *c* (prepared by reduction of cytochrome with NaBH_4_ and HCl) at *λ* = 550 nm with 580 nm as the reference wavelength (*ε* = 19.1 mM^−1 ^cm^−1^). The activities of the mitochondrial respiratory chain complexes were expressed as nmol/min^−1^/mg of protein^−1^.

### 2.7. Statistical Analysis

In the present study, the hypothesis is that molecular biomarkers are affected by the following factors: (1) age: young versus middle-aged and (2) training intensity: nontrained versus 0.8 km/h speed versus 1.2 speed km/h. The results about the descriptive characteristics of young and middle-aged rats before exercise protocols were expressed as mean and standard error median (SEM) and were evaluated using the unpaired Student's *t*-test. While the results about the western blot analyses were expressed as the mean area of the apparent band ± SEM (arbitrary units were calculated as area versus density), the activity of Krebs cycle enzymes and the activity of mitochondrial respiratory chain enzymes were expressed as nmol/min/mg of protein ± SEM. Differences between the groups for the mentioned parameters were evaluated using two-way analysis of variance (ANOVA) followed by the Bonferroni* post hoc* test. A probability of less than 0.05 was considered to be significant. The software used for the analysis of the data was the Statistical Package for the Social Sciences (SPSS) version 16.0 for Windows.

## 3. Results 

### 3.1. Descriptive Characteristics of Young and Middle-Aged Rats before Exercise Protocols

According to Table 1, the middle-aged rats presented higher values of body weight (526 ± 12.31 versus 218.9 ± 10.02 g), epididymal fat (3.9 ± 0.4 versus 1.2 ± 0.2 g/100 g), and serum insulin (4.2 ± 0.7 versus 1.3 ± 0.5 ng/mL) compared to young rats.

### 3.2. TNF-*α*, IL-1*β*, and NF-*κ*B Protein Levels in Quadriceps of Young and Middle-Aged Rats after Exercise Training at 0.8 and 1.2 km/h

The protein levels of TNF-*α*, IL-1*β*, and NF-*κ*B were higher in the quadriceps of middle-aged NE compared to young NE rats (Figures 1(a)–1(c)). Both groups (i.e., young and middle-aged rats) were trained at 0.8 km/h which decreased the protein levels of TNF-*α*, IL-1*β*, and NF-*κ*B compared to their respective NE groups; however, the middle-aged rats presented higher protein levels of TNF-*α*, IL-1*β*, and NF-*κ*B compared to young rats at the 0.8 km/h training intensity (Figures 1(a)–1(c)). In addition, both groups were trained at 1.2 km/h which decreased the protein levels of TNF-*α*, IL-1*β*, and NF-*κ*B compared to their respective 0.8 km/h groups, but no differences were observed between young and middle-aged rats at the 1.2 km/h training intensity (Figures 1(a)–1(c)). *β*-actin protein levels were similar between the groups (Figures 1(a)–1(c)—lower panels).

### 3.3. SIRT-1 and PGC-1*α* Protein Levels and AMPK and ACC Phosphorylation in Quadriceps of Young and Middle-Aged Rats after Exercise Training at 0.8 and 1.2 km/h

We evaluated pivotal molecules involved in mitochondrial function and oxidative metabolism. While AMPK phosphorylation decreased in the quadriceps of middle-aged NE compared to young NE rats (Figure 2(a)), no significant differences were observed between these groups (i.e., young and middle aged rats) at NE situation for ACC phosphorylation (Figure 2(b)). Both groups (i.e., young and middle-aged rats) were trained at 0.8 km/h which increased AMPK and ACC phosphorylations compared to their respective NE groups; however, the middle-aged rats presented lower AMPK and ACC phosphorylations compared to the young rats at the 0.8 km/h training intensity. In addition, both groups were trained at 1.2 km/h which increased the AMPK and ACC phosphorylation compared to their respective 0.8 km/h groups, but no differences were observed between young and middle-aged rats at the 1.2 km/h training intensity (Figures 2(a) and 2(b)). Total AMPK and ACC protein levels were similar between the groups (Figures 2(a) and 2(b)—lower panels).

SIRT-1 and PGC-1*α* protein levels decreased in the quadriceps of middle-aged NE rats compared to young NE rats (Figures 2(c) and 2(d)). Both groups (i.e., young and middle-aged rats) were trained at 0.8 km/h which increased the protein levels of SIRT-1 and PGC-1*α* compared to their respective NE groups; however, the middle-aged rats presented lower protein levels of SIRT-1 and PGC-1*α* compared to young rats at the 0.8 km/h training intensity. In addition, both groups were trained at 1.2 km/h which increased the protein levels of SIRT-1 and PGC-1*α* compared to their respective 0.8 km/h groups, but no differences were observed between young and middle-aged rats at the 1.2 km/h training intensity (Figures 2(c) and 2(d)).

### 3.4. CPT1, Cyt-C, and SDH Protein Levels and SDH and Citrate Synthase Activities in Quadriceps of Young and Middle-Aged Rats after Exercise Training at 0.8 and 1.2 km/h

Subsequently, we determined the protein levels and activities of important metabolic enzymes. Lower protein levels of CPT1 and Cyt-c were observed in the quadriceps of middle-aged NE rats compared to young NE rats. Both groups (i.e., young and middle-aged rats) were trained at 0.8 km/h which increased the protein levels of CPT1 and Cyt-c compared to their respective NE groups; however, the middle-aged rats presented lower protein levels of CPT1 and Cyt-c compared to young rats at the 0.8 km/h. In addition, both groups were trained at 1.2 km/h which increased the protein levels of CPT1 and Cyt-c compared to their respective 0.8 km/h groups, but no differences were observed between young and middle-aged rats at the 1.2 km/h training intensity (Figures 3(a) and 3(b)). The SDH protein levels did not present significant differences between young and middle-aged rats for the studied experimental situations (i.e., NE, 0.8 and 12 km/h; Figure 3(c)). The SDH activity was not different between young and middle-aged rats for the NE situation. The young rats were trained at 0.8 km/h which increased the SDH activity compared to their respective NE group. On the other hand, SDH activity was lower in middle-aged rats compared to young rats at the 0.8 km/h training intensity. In addition, middle-aged rats were trained at 1.2 km/h which increased the SDH activity compared to their respective 0.8 km/h group, but no significant differences were observed between young and middle-aged rats at the 1.2 km/h training intensity (Figure 3(d)).

The protein levels and activity of citrate synthase were lower in the quadriceps of middle-aged NE rats compared to young NE rats. Both groups (i.e., young and middle-aged rats) were trained at 0.8 km/h which increased the protein levels of citrate synthase compared to their respective NE groups; however, the middle-aged rats presented lower protein levels and activity of citrate synthase compared to young rats at the 0.8 km/h. In addition, both groups were trained at 1.2 km/h which increased the protein levels and activity of citrate synthase compared to their respective 0.8 km/h groups, but no differences were observed between young and middle-aged rats at the 1.2 km/h training intensity (Figures 3(e) and 3(f)).

### 3.5. Mitochondrial Complexes Activities in Quadriceps in Young and Middle-Aged Rats after Exercise Training at 0.8 and 1.2 km/h

The young and middle-aged rats did not present significant alterations for the complexes I, II, and II-III activities at the NE and 0.8 km/h situations. However, the young and middle-aged rats were trained at 1.2 km/h which increased the complexes I, II, and II-III activities compared to their respective 0.8 km/h groups. In addition, for these complexes, we did not observe significant differences between young and middle-aged rats at the 1.2 km/h training intensity (Figures 4(a)–4(c)). The complex II activity was higher in young rats compared to middle-aged rats at the 0.8 km/h training intensity (Figure 4(b)). The complex IV activity decreased in the quadriceps of middle-aged NE rats compared to young NE rats. The young rats were trained at 0.8 km/h which increased the complex IV activity compared to their respective NE group. The complex IV activity of the middle-aged rats was lower compared to young rats at the 0.8 km/h training intensity. In addition, both groups (i.e., young and middle-aged rats) were trained at 1.2 km/h which increased the complex IV activity compared to their respective 0.8 km/h groups, but no differences were observed between young and middle-aged rats at the 1.2 km/h training intensity (Figure 4(d)).

## 4. Discussion

The main findings of the present investigation are (a) the aging process is associated with the increase of TNF-*α*, IL-1*β*, and NF-*κ*B protein levels and with the decrease of the AMPK phosphorylation and SIRT-1 and PGC-1*α* protein levels; (b) the young and middle-aged rats were trained at 0.8 km/h which decreased the TNF-*α*, IL-1*β*, and NF-*κ*B protein levels and increased the AMPK phosphorylation and SIRT-1 and PGC-1*α* protein levels compared to their respective NE groups, although the young rats presented lower values (for TNF-*α*, IL-1*β*, and NF-*κ*B) and higher values (for SIRT-1, PGC-1*α*, and AMPK) compared to the middle-aged rats inside this specific training intensity; (c) the young and middle-aged rats were trained at 1.2 km/h which decreased the TNF-*α*, IL-1*β*, and NF-*κ*B protein levels and increased the AMPK phosphorylation and SIRT-1 and PGC-1*α* protein levels compared to their respective 0.8 km/h groups; (d) interestingly, at this training intensity (i.e., 1.2 km/h), the behavior of the analyzed molecules was not different between young and middle-aged rats.

The inflamm-aging process is associated with high levels of TNF-*α*, IL-1*β*, and NF-*κ*B in skeletal muscle of elderly individuals and rodents [23, 30]. The present results are in accordance with Della Gata et al. [23] showing that exercise training is able to revert partially the high levels of cytokines induced by the inflamm-aging process. On the other hand, up to today, this is the first investigation showing that high training intensities lead to better responses of TNF-*α*, IL-1*β*, and NF-*κ*B in skeletal muscle of middle-aged rats. These responses may be linked to the increases observed in the protein levels of PGC-1*α*, once this molecule acts as a suppressor of inflammatory cytokines [24].

Aging process is associated with the reduction of the muscle functionality that, at least in part, is linked to mitochondrial dysfunction [1, 31–34]. Some studies have shown that key molecules are involved in this process, such as SIRT-1, AMPK, and PGC-1*α* [9–12, 22, 32]. The role of SIRT-1 in skeletal muscle is mainly attributed to its ability to deacetylate and activate PGC-1*α* [9, 12, 22]. PGC-1*α* orchestrates the genetic program that allows skeletal muscle cell adaptation to meet the energy demands. Ectopic expression of PGC-1*α* in myotubes increases the respiratory chain gene expression (i.e., cytochrome c) and promotes mitochondrial biogenesis [12]. Furthermore, it is well known that AMPK upregulates SIRT-1 activity in skeletal muscles [21, 35]. The AMPK activity inhibition prevents the deacetylation of PGC-1*α* by SIRT-1 in skeletal muscle cells in response to glucose deprivation, decreasing the mitochondrial complex activity and damaging the fatty acid oxidation metabolism [21, 35]. In addition, the study of AMPK deficient mice evidenced the impairment of PGC-1*α* deacetylation in correlation with a failure of muscle metabolism adaptation in response to exercise [21, 35].

Thus, in the present investigation, we tested the hypothesis that high training intensity is more effective than low training intensity in restoring SIRT-1, AMPK, PGC-1*α*, and related metabolic enzymes that decrease with aging. In summary, these molecules increased when the experimental groups were trained at 0.8 km/h (i.e., compared to their respective NE groups) and at 1.2 km/h (i.e., compared to their respective 0.8 km/h groups). In addition, these molecules were higher in young rats compared to middle-aged rats at the 0.8 km/h training intensity but were not different at the 1.2 km/h training intensity. These findings suggest that middle-aged rats will present the same molecular responses as young rats when the training intensity is high. In accordance with the elegant study of Koltai et al. [6], we demonstrated that treadmill training may reverse the negative effects of aging on pivotal molecules that are associated with the mitochondrial control of skeletal muscle of rats. In fact, Koltai et al. [6] also verified that treadmill training increased the SIRT-1 activity in both young and aged rats (26 months of age).

The elegant study of Cantó et al. [35] showed that AMPK activation precedes and determines the changes in SIRT-1 activity in situations of energy stress. The regulation of the acetylation levels of transcriptional regulators through the AMPK/SIRT-1 axis provides a mechanism by which mitochondrial and lipid oxidation genes can be rapidly and selectively controlled in response to energy levels [21, 34, 36]. In the present investigation, we observed that the phosphorylation of AMPK and the protein levels of SIRT-1 and PGC-1*α* decreased in the quadriceps of NE middle-aged rats compared to the NE young rats. On the other hand, these proteins increased when the experimental groups were trained at 0.8 km/h compared to their respective NE groups, although the results of the young rats were higher compared to the middle-aged rats at 0.8 km/h training intensity. However, these proteins remained unchanged between young and middle-aged rats at 1.2 km/h training intensity. Tobina et al. [24] cited that AMPK is activated by the decrease in the ATP/AMP ratio and phosphocreatine (CP) and glycogen levels. On the other hand, the CP and glycogen depletion are dependent on the exercise intensity [37, 38]. Although we did not measure the CP and glycogen concentrations in the present paper, it is possible to hypothesize that the higher training intensity led to higher depletion of these substrates and was responsible for the higher AMPK activation.

Similar results were observed for CPT1 and Cyt-c protein levels. Interestingly, Suwa et al. [39] observed that the protein expressions of SIRT-1 but not PGC-1*α* increased in response to training. The differences between our data and the results of Suwa et al. [39] may be related to the differences in the exercise protocols and age of the studied rats. Aging process may impair the oxidative capacity of skeletal muscles [33]. The mitochondrial respiratory chain is composed of four respiratory complexes (complexes I–IV), and each one is capable of catalyzing electron transfers in a partial reaction of the respiratory chain. It is known that citrate synthase and succinate dehydrogenase activities can be used to estimate mitochondrial content [40] and mitochondrial complexes can reflect the mitochondrial oxidative capacity. In accordance with the results of AMPK phosphorylation, SIRT-1 and PGC-1*α* protein levels, the activity and protein levels of citrate synthase, and the activities of the mitochondrial complexes I, II, II-III, and IV also increased in both groups (i.e., young and middle-aged rats) at the 1.2 km/h training intensity.

Studying AMPK knockout mice, Jørgensen et al. [41] reported significant reductions in mitochondrial markers (i.e., citrate synthase activity and protein contents of one or more complexes in the mitochondrial respiratory chain). On the other hand, SIRT-1 played a crucial role in the ability of AMPK increasing the mitochondrial respiration, once the long-term AICAR effects on cellular oxygen consumption were blunted by knocking-down SIRT-1 [35]. In addition, the authors also observed a decrease in the lipid oxidation and an increase in alternative substrate oxidation [35]. In fact, the direct oleate oxidation measurement confirmed that the AICAR chronic effects on lipid oxidation were blunted in myotubes when the SIRT-1 expression was knocked down [35]. Therefore, the AMPK and SIRT-1 signaling pathways have similar effects on lifespan, aging, and metabolism. Like SIRT-1, AMPK has been considered as one of several molecules involved in the mammalian longevity regulation [42].

Other investigations have verified the training effects on the current studied parameters in aged rats [22, 43]. For example, Ljubicic and Hood [44] examined a very extreme form of muscle activation, chronic electrical stimulation, in rats (i.e., 36 months of age), and they verified that the mitochondrial biogenesis signaling response was compromised. These data indicate that high exercise intensity (or muscle activation) in aged rats is not sufficient to correct the age-related decline in the muscle aerobic plasticity. Recently, Bayod et al. [22] observed that treadmill training during 36 weeks increased the protein content and activity of SIRT-1 and the protein expression of PGC-1*α* in the heart, muscle, and liver of aged rats. However, no changes in AMPK activation or mitochondrial biogenesis were found after 36-week treadmill training.

The aging process is associated with the decline of both AMPK and SIRT-1 activities. For example, the AMPK activation by AICAR or exercise is blunted in skeletal muscles of old rats (i.e., 28 months of age). Furthermore, the mitochondrial biogenesis was also reduced after chronic activation of AMPK with *α*-guanidinopropionic acid (*α*-GPA) [19]. On the other hand, SIRT-1 protein levels are diminished in mouse embryonic fibroblasts that exhibit premature senescence [45]. However, as previously mentioned, there is a considerable variability of aging impact on mitochondrial function [2–6]. The different types of studied rodents, their respective aging phases, and the analyzed parameters may be considered by the discrepancies mentioned above, justifying the new investigations to elucidate the relationship between aging and its molecular consequences. In addition, the selection of middle-aged rats to study molecular and physiological changes related to mitochondrial function is justified because this life period still allows the use of preventive actions that can lead to healthy aging.

In summary, we conclude that age-related increases in TNF-*α*, IL-1*β*, and NF-*κ*B and age-related declines in the phosphorylation of AMPK and in the protein levels of SIRT-1 and PGC-1*α* in skeletal muscle can be reversed and largely improved by treadmill exercise training. In addition, the present data demonstrated that to achieve changes in muscle of middle-aged rats that are similar to young rats, high training intensities are necessary.

## Figures and Tables

**Figure 1:** Effects of exercise protocols performed in different intensities on the TNF-*α*, IL-1 *β*, and NF-*κ*B protein levels in the quadriceps of young and middle-aged rats. Protein levels of TNF-*α* (a), IL-1*β* (b), and NF-*κ*B (c). Upper panels show representative blots of these proteins. Lower panels show representative blots of *β*-actin (a)–(c) protein levels. The results of scanning densitometry are expressed as arbitrary units. Bars represent means ± SEM of six rats. *P < 0.05 versus young NE rats, ^#^ *P* < 0.05 versus middle-aged NE rats, ^$^ *P* < 0.05 versus young rats at 0.8 km/h, and ^&^ *P* < 0.05 versus middle-aged rats at 0.8 km/h.

**Figure 2:** Effects of exercise protocols performed in different intensities on the AMPK and ACC phosphorylation and SIRT-1 and PGC-1*α* protein levels in the quadriceps of young and middle-aged rats. Phosphorylation of the AMPK (a) and ACC (b) and protein levels of SIRT-1 (c) and PGC-1*α* (d). Upper panels show representative blots of these proteins. Lower panels show representative blots of total AMPK (a) and total ACC (b) protein levels. The results of scanning densitometry are expressed as arbitrary units. Bars represent means ± SEM of six rats. *P < 0.05 versus young NE rats, ^#^ *P* < 0.05 versus middle-aged NE rats, ^$^ *P* < 0.05 versus young rats at 0.8 km/h, and ^&^ *P* < 0.05 versus middle-aged rats at 0.8 km/h.

**Figure 3:** Effects of exercise protocols performed in different intensities on the CPT1, Cyt-c, citrate synthase, and SDH protein levels and SDH and citrate synthase activity in the quadriceps of young and middle-aged rats. Protein levels of CPT1 (a), Cyt-c (b), SDH (c), and citrate synthase (e). Upper panels show representative blots of these proteins. The results of scanning densitometry are expressed as arbitrary units. The activities of succinate dehydrogenase (d) and citrate synthase (f) are expressed as nmol/min/mg of protein. Bars represent means ± SEM of six rats. *P < 0.05 versus young NE rats, ^#^ *P* < 0.05 versus middle-aged NE rats, ^$^ *P* < 0.05 versus young rats at 0.8 km/h, and ^&^ *P* < 0.05 versus middle-aged rats at 0.8 km/h.

**Figure 4:** Effects of exercise protocols performed in different intensities on the complexes I, II, II-III, and IV activities in the quadriceps of young and middle-aged rats. Complexes I (a), II (b), II-III (c), and IV (d) activities are expressed as nmol/min/mg of protein. *P < 0.05 versus young NE rats, ^#^ *P* < 0.05 versus middle-aged NE rats, ^$^ *P* < 0.05 versus young rats at 0.8 km/h, and ^&^ *P* < 0.05 versus middle-aged rats at 0.8 km/h.

**Table 1:** Descriptive characteristics of young and middle-aged rats (*n* = 8) before exercise protocols expressed as mean ± SEM.

Parameters	Young rats	Middle-aged rats
	(*n* = 8)	(*n* = 8)
Body weight (g)	218.9 ± 10.02	526 ± 12.31*
Epididymal fat (g/100 g)	1.2 ± 0.2	3.9 ± 0.4*
Serum insulin (ng/mL)	1.3 ± 0.5	4.2 ± 0.7*
Blood glucose (mg/dL)	87.7 ± 7.54	92.9 ± 6.92

*P < 0.05 significant difference versus young rats.
